This article has been retracted.

# Sports Medical Image Modeling of Injury Prevention in Wushu Training

**DOI:** 10.1155/2022/5201952

**Published:** 2022-08-09

**Authors:** Yuanyuan Feng

**Affiliations:** ^1^Faculty of History and Culture, Chengdu Sport University, Chengdu, Sichuan 610041, China; ^2^College of Physical Education, Sichuan Agricultural University, Ya'an, Sichuan 625014, China

## Abstract

In order to solve the problem of injury prevention in Wushu training, this paper proposes a research on modeling using sports medical images. The main content of this technology research is to drive the muscle strength modeling method based on the sports medical image data. According to the acquisition of MRI/CT images, through the research and application of DFIS, it is concluded that the research on sports medical image modeling has a high accuracy for injury prevention in Wushu training. The experimental results show that translation accuracy ≤ 0.03~0.27, rotation accuracy ≤ 0.24~0.63, flexion and extension accuracy ≤ 0.1, translation retest error ≤ 0.2~1.2, rotation retest error ≤ 0.5~3.4, rotation retest accuracy ≤ 0.4~1.04, and sports medical images have a high accuracy for injury prevention in Wushu training. It is proved that the research on sports medical image modeling is effective and accurate for the problem of injury prevention in Wushu training.

## 1. Introduction

In the process of the steady development of China's sports cause, the social and economic developments are striding forward, the development of Wushu is also moving forward, and its movement difficulty is also gradually increasing, resulting in many Wushu Athletes' increasing injuries in training [1]. Athletes' injuries will not only make their bodies bear some degree of pain but also affect their future training and even affect the psychology of Wushu athletes. Therefore, in the development process of Wushu events, we should constantly summarize and summarize various influencing factors of athletes' sports injury, record various morbidity laws, and take effective measures to prevent according to specific reasons, so as to effectively reduce the probability of athletes' injury and improve the efficiency of Wushu events, so as to promote the orderly development of Wushu.

Compared with other sports, Wushu is more confrontational. Athletes must master the corresponding movement skills before they can complete the confrontational training more easily and freely. In the teaching and training of Wushu, sports personnel will be free from sports injuries of different degrees, which will also have an impact on the physical and mental health of sports personnel. Therefore, in Wushu teaching and training, teachers must take scientific measures to prevent and deal with injury accidents in combination with the actual situation, so that athletes can learn Taekwondo knowledge and skills more happily. Sports injury refers to the injury occurring in the process of sports. It is closely related to sports events, sports technical actions, physical conditions of exercisers, venues, and equipment. If the method of engaging in sports activities is improper, it may cause unnecessary harm and bring adverse effects on everyone's physical health, study, life, and psychology. Sports injuries are common among athletes, who need to regularly carry out various sports, and require high technical difficulty, high intensity, and strong antagonism, so the incidence of sports injuries is higher [2].

In recent years, Wushu has developed rapidly in various provinces and cities, is popular widely, and is welcomed and loved by the masses. However, at the same time of sports, because people have not yet fully mastered and understood Wushu, there are hidden dangers in the training process, and injuries often occur [3]. Therefore, corresponding preventive measures should be put forward in time and effectively to effectively ensure the performance and physical health in Wushu training.

## 2. Literature Review

With the vigorous development of physical education in the country, under the current background, physical education has gradually developed to lifelong physical education. Lifelong physical education pursues the continuous physical exercise and the improvement of physical learning ability in people's life. It is a new concept accompanied by the importance of lifelong learning. The implementation of lifelong physical education in sports will bring about great changes in the concept of physical education teaching and training [4]. As an important part of physical exercise theory, the prevention mechanism of sports injury is closely related to people's physical health, the effective implementation of physical education teaching and training, and the improvement of lifelong exercise ability. Therefore, the content of the research on the prevention mechanism of sports injury itself is also an important part of lifelong physical education, which may be closely connected with the teaching content of its related courses. Therefore, considering the particularity of sports and the requirements of lifelong physical education, the research on the prevention mechanism of sports injury has high practical value. We should strengthen the monitoring of exercise load, reasonably arrange teaching and training, take preventive measures, reasonably arrange teaching and training, formulate training plans in line with scientific principles, and scientifically and reasonably arrange preparatory activities. The purpose of preparatory activities is to improve the excitability of the central nervous system through a variety of exercises, enhance the coordination ability of various organ systems, overcome the inertia of human body functions, and enable the human body to be prepared from a relatively static state to a tense active state, so as to shorten the adaptation process of the human body to movement. Generally speaking, the injuries caused in the process of Wushu training are caused by the ideological neglect of athletes and Wushu coaches. In particular, they attach great importance to the training results but neglect the safety education. Therefore, they do not give relevant reminders to athletes and do not use useful measures to carry out corresponding prevention. Some athletes do not pay attention to their own safety issues in the process of Wushu training, and their attitude is not correct, which greatly increases the probability of physical injury. In a word, it is very important to pay attention to the prevention and treatment of athletes' sports injuries in Wushu training. Therefore, in practice, we must fully understand the common injuries in Wushu training, grasp the causes of injuries, and take scientific measures to prevent sports injuries on this basis, so as to promote the quality of Wushu training.

In view of the above problems, this paper proposes a research on sports medical image modeling to improve injury prevention in Wushu training [5]. The main content of this technology research is to drive the muscle strength modeling method based on the sports medical image data. According to the acquisition of MRI/CT images, through the research and application of DFIS, it is concluded that the research on sports medical image modeling has a high accuracy for injury prevention in Wushu training. So as to provide more accurate data, more advanced technology and more reliable methods [6].

## 3. Research Methods

### 3.1. Data Driven Muscle Strength Modeling Method for Sports Medical Images

#### 3.1.1. Modeling Method and Process

The data-driven modeling process of sports medical images includes the following steps, as shown in Figure 1: the first is the acquisition of medical image data, usually including CT or MRI. The second is the registration, fusion, and segmentation of the acquired medical image data. Then, the three-dimensional reconstruction of the target area is carried out, and the physical parameters such as the volume and moment of inertia of the current area are calculated. Then, the joint system is modeled. Mechanical modeling of skeletal muscle was based on hill theory. Then, the kinematics data and inverse dynamics data are used for multibody dynamics modeling and analysis [7]. Finally, the static optimization method is used to estimate the muscle force, and the fusion analysis of the model is carried out.

#### 3.1.2. Acquisition of MRI/CT Images

Both MRI and CT are indispensable medical imaging techniques in clinic. Because of the difference between MRI and CT images, the fusion of MRI and CT images becomes very meaningful. The first step of image fusion is registration. Segmentation is to generate pixel set (pixel block) from the image containing the target tissue part and separate it from the whole image. In medical images, segmentation is usually related to the specific structure described. The segmentation algorithm of medical images combines the data structure and medical information and achieves the purpose of target tissue segmentation through the combination of the two. Fusion is to extract the information of interest from the image data from different sources and then combine it into a new image that can reflect the characteristics of a variety of image data [8].

The three-dimensional reconstruction of the target area and the complete three-dimensional curve and surface geometric model are the basis of the human biomedical simulation model and subsequent dynamic analysis and calculation [9]. In this paper, the cubic rational periodic B-spline curve approximation method is used to segment the fused image directly and output the spline curve model of bone tissue contour directly. This algorithm has the following advantages: firstly, with the help of anatomists, accurate segmentation results can be obtained; Secondly, by using the local property of cubic rational periodic B-spline curve, the curve shape can be easily adjusted, and at the same time, a very accurate approximation curve can be obtained with only a small number of feature points. The final data can be written in IGES format, which is a standard three-dimensional model data file for subsequent skeletal muscle force calculation and analysis.

#### 3.1.3. Medical Imaging Technology

The rapid development of medical imaging technology, computer image processing technology, and network technology has promoted the continuous upgrading of radiotherapy equipment used in clinical treatment [10]. After the arrival of the era of precision radiotherapy, three-dimensional conformal radiotherapy, spiral tomography, and X-ray real-time imaging technology have been applied in the field of clinical treatment. In terms of the current development of clinical treatment, medical image 3D reconstruction technology plays an important role in the treatment planning system. Registration between two-dimensional images and three-dimensional models is inseparable from the support of three-dimensional reconstruction of medical images. CT diagnosis is a common technique in clinical treatment. It is a reference factor for medical staff to judge the condition and determine the treatment plan. At this stage, China has entered the digital imaging era. The accuracy of diagnostic basis is the focus of clinical treatment [11].

During the study, retrospective analysis was conducted according to the diagnosis of patients. During the study, the test verification platform included X-ray machine, graphic workstation, operating table, and other equipment. According to the actual situation of the experimental study, the relevant personnel used CT equipment to complete the bone information scanning and input the relevant image data into the workstation. In the three-dimensional model and processing stage, the researchers used image noise reduction, threshold division, and isoline extraction to carry out image preprocessing and determine the closed isoline of each image in the CT data. The method used in the construction of the 3D model is volume rendering algorithm [12].

In the process of 3D model construction, relevant personnel used image noise reduction measures to remove the noise in CT image data and improve image quality. During modeling, image segmentation tools are used as image segmentation algorithms. During the implementation of 3D reconstruction of CT data, relevant personnel realized 3D image surface by means of surface rendering and volume rendering [13]. The fitting curve of positive-position mutual information value is shown in Figure 2. In this fitting curve, there are two extreme values in the mutual information curve.

The lateral fitting curve of the patient's CT image processing results is shown in Figure 3. According to the contents of the figure, the lateral fitting curve only contains an extreme value. Researchers can obtain complete 2D-3D registration parameters according to the research methods applied to this study [14].

### 3.2. Research and Application of DFIS

#### 3.2.1. DFIS Study

DFIS originated from the fluoroscopy imaging technology invented in 1895 [15]. Since its invention, fluoroscopy imaging technology has been widely used in medical imaging detection because of its penetrability and noninvasiveness. However, medical imaging detection is mainly based on static image analysis, which has great limitations in the field of human motion. Therefore, researchers have combined fluoroscopy imaging technology with image shooting technology to invent a single plane fluoroscopy analysis system, which has been widely used in the field of medicine and human low-speed movement. Its limitation is that it is unable to quantify the 6DOF movement of joint bone structure and accurately analyze the relationship between the movement of bone structure and injury. Combining fluoroscopy imaging technology, 2D/3D registration technology, and 3D motion analysis technology, a low-speed DFIS (sampling frequency ≤ 30 Hz) is developed to realize dynamic 3D tracking and analysis of bone and joint motion in vivo 2-25. The biplane orthogonal fluorescence imaging system is improved to expand the shooting range and increase the shooting frequency (sampling frequency ≥ 100 Hz, shutter speed ≥ 1/500 s). At present, these systems have been successfully applied in the fields of cardiac/cerebral angiography imaging, joint surgery positioning, personalized 3D joint prosthesis replacement, and the movement of human bone structure in the body weight-bearing functional position.

Human movement takes the bone as lever, the joint as fulcrum, and the skeletal muscle contraction as power. The mechanism of joint injury (usually caused by irregular movement or high impact) has always been a research hotspot [16]. The commonly used traditional motion capture system indirectly measured the rotation angle error of subtalar joint more than 10°. The tibial movement distance during knee flexion is greater than the real movement distance. Due to the error of the skin and soft tissue, there is a defect in indirect inference when discussing the mechanism of joint injury. DFIS can dynamically track the position relationship and deformation of joint bone structure, ligament, and cartilage in vivo during human movement and, more intuitively, truly and accurately explore the mechanism of joint injury. Researchers have successfully used DFIS to explore some sports injury mechanisms of shoulder joint, lumbar spine, knee joint, and ankle joint (the knee joint is the most concerned), and there are still many sports injury mechanisms that have not been explored [17].

#### 3.2.2. Application of DFIS in the Mechanism of Knee Joint Sports Injury

Some studies have used DFIS to explore the mechanism of anterior cruciate ligament (ACL) injury caused by weight-bearing knee bending and landing. The results showed that the peak value of relative elongation of posterior lateral bundle (PL) of ACL was 5.9% when the subjects bent the knee 15° with load, and the peak value of relative elongation of anterior medial bundle (AM) of ACL was 4.4% when the subjects bent the knee 30° with load, indicating that the pl of ACL was easy to break when the subjects bent the knee 15° with load. The AM of the ACL is prone to fracture at 30 flexion. The study also found that the peak distance of tibial displacement at 40 cm landing was 5.6 mm, which was greater than 3.1 mm when walking (90 steps/min) and 2.6 mm when stretching the knee without load. There was no difference in the peak value of tibial internal rotation at 40 cm landing, maximum isometric knee extension (flexion 70°), and no load extension (14.5°~19.4°), which was greater than 3.907 when walking. It indicates that the increase of applied load will increase the distance of tibial femoral forward movement and then increase the risk of ACL fracture. This situation is related to the increase of exercise height and intensity and the increase of muscle and soft tissue load. When the healthy subjects landed with straight knee and bent knee, there was no significant difference in the peak value of tibial femoral forward movement distance, but the ground reaction force and knee extension torque on the straight knee landing were greater than those on the bent knee landing. The passive relaxation of the knee joint forward was related to the peak value of tibial forward movement distance at the landing time. The tibial anteroposterior movement distance of healthy subjects was not related to knee extension torque or anteroposterior shear force 3.51, indicating that joint relaxation may increase the risk of ACL injury when landing. When the subject lands, the knee valgus angle has a direct relationship with the tibial forward displacement distance and lateral displacement distance. It indirectly indicates that the increase of knee valgus may increase the risk of ACL injury [18].

Some studies have used DFIS to discuss the mechanism of knee medial cartilage injury caused by weight-bearing flexion, walking, and stepping on steps. The results show that the probability of knee osteoarthritis is twice that of ordinary people, and the pressure behind the knee joint is 58.3% higher than that of daily walking. From full extension to 90° flexion, the contact point of the tibia and femur is at the medial side of tibial plateau and femoral condyle. The contact point between tibia and femur platform was more medial and lateral in large-scale flexion. The minimum deformation of knee joint cartilage occurs when the knee is bent by 30°, and the maximum deformation occurs when the knee is bent by 120°, and the contact area and deformation of the medial side (see Figure 4) are greater than that of the lateral side (see Figure 5) indicating that the posterior pressure in the tibial plateau is large during the large-scale flexion of the knee joint. If the knee is bent by more than 120° for a long time, the incidence of medial cartilage damage increases. The study found that when the subjects were treading on the ground at a slow pace (knee extension), the horizontal range of motion of the medial femoral condyle was greater than that of the lateral femoral condyle. When stepping on the steps to extend the knee, the contact point between the femur and the medial tibial plateau moved backward. The contact radius of the medial tibial plateau in the sagittal plane is larger than that of the lateral tibial plateau, indicating that the pedaling and stretching exercise will increase the injury rate of the medial femoral cartilage and the medial tibial plateau of the knee joint. Therefore, repeated large-scale flexion and pedaling and stretching of the knee joint may cause damage to the medial cartilage of the knee joint [19].

## 4. Result Analysis

The application of DFIS in sports medicine depends on the reliability, validity, and accuracy of the system in analyzing 6DOF motion of human joint internal structure [20]. Tantalum beads were implanted into human humerus, scapula, clavicle, and lumbar vertebrae. Steel balls were implanted into human lumbar vertebrae and medullary joints. Balls of different materials were implanted into the knee joint specimens. The specimens of the tibia, talus, and calcaneus were embedded with copper beads [21]. The foot model and gait are used to simulate the robot, and the model is used to calculate. It is confirmed that the system can be used to analyze the 6DOF constant and high-speed movements of the internal bone structures of shoulder, lumbar spine, medullary joint, knee, and ankle and has certain effectiveness, repeatability, and accuracy, as shown in Table 1. It is concluded that the translation accuracy is ≤0.03~0.27, the rotation accuracy is ≤0.24~0.63, the flexion and extension accuracy is ≤0.1, the translation retest error is ≤0.2~1.2, the rotation retest error is ≤0.5~3.4, and the rotation retest accuracy is ≤0.4~1.04.

## 5. Conclusion

In order to solve the problem of injury prevention in Wushu training, this paper presents a research on modeling using sports medical images. The main content of this technology research is to drive the muscle strength modeling method based on the sports medical image data. According to the acquisition of MRI/CT images, through the research and application of DFIS, it is concluded that the research on sports medical image modeling has a high accuracy for injury prevention in Wushu training. This paper discusses the potential risk factors and possible injury mechanism of joint injury in a deeper level, which can provide more accurate data, more advanced technology, and more reliable methods for the standardization of movement, the accurate diagnosis and treatment of sports injury, the formulation of personalized rehabilitation plan, and the development of sports protective equipment.

## Figures and Tables

**Figure 1:** Flow chart of muscle strength modeling driven by medical image data.

**Figure 2:** Positive fitting curve.

**Figure 3:** Lateral fitting curve.

**Figure 4:** Contact area and track of femur and tibial cartilage.

**Figure 5:** Contact area and track between tibia and medial and lateral femoral condyle cartilage.

**Table 1:** Reliability, validity, and accuracy of DFIS in evaluating human joint motion.

	Translation accuracy (mm)	Rotation accuracy (°)	Flexion and extension accuracy (°)	Translation retest error (mm)	Rotation retest error (°)	Rotation remeasurement accuracy (°)
Meng brachial joint	≤0.13~0.39	≤0.47~0.7	—	≤0.2~1.2	—	—
Acromioclavicular joint	—	—	—	—	≤0.5~3.4	≤0.4~1.04
Lumbar vertebra	≤0.35~0.43	≤0.65~0.7	—	≤0.36	—	—
Brittle joint	≤0.2	≤0.45~0.59	—	—	—	—
Knee joint	≤0.15	—	≤0.1	—	—	—
Ankle joint	≤0.03~0.27	≤0.24~0.63	—	—	—	—

## Data Availability

The data used to support the findings of this study are available from the corresponding author upon request.
